The article "miR‐944 inhibits metastasis of gastric cancer by preventing the epithelial–mesenchymal transition via MACC1/Met/AKT signaling" was retracted in 2022. Reasons: duplicated images; signs of a paper mill.

# miR‐944 inhibits metastasis of gastric cancer by preventing the epithelial–mesenchymal transition via MACC1/Met/AKT signaling

**DOI:** 10.1002/2211-5463.12215

**Published:** 2017-05-24

**Authors:** Tao Pan, Wenjun Chen, Xiaoming Yuan, Jun Shen, Chuan Qin, Linbo Wang

**Affiliations:** ^1^ Department of Surgical OncologySir Run Run Shaw HospitalSchool of MedicineZhejiang UniversityHangzhouChina

**Keywords:** EMT, gastric cancer, MACC1, Met/AKT signaling, microRNA‐944

## Abstract

MicroRNAs (miRNAs) are reported to play vital roles in tumor progression. Recently, miR‐944 was reported to play either an oncogenic or tumor suppressive role in human cancers. However, the expression of miR‐944 and its exact role in gastric cancer (GC) remain unknown. This study aimed to evaluate whether loss of miR‐944 could promote the epithelial–mesenchymal transition (EMT) of GC. Reduced expression of miR‐944 was identified in 40 pairs of human GC and matched normal tissues by qRT‐PCR. Reduced expression of mi‐944 was also observed in GC cell lines. Restoration of miR‐944 inhibited cell migration and invasion in MGC‐803 cells, while its loss facilitated metastasis of SGC‐7901 and BGC‐823 cells. Notably, miR‐944 overexpression prohibited EMT of GC cells *in vitro*, while miR‐944 knockdown had the opposite effect. Bioinformatics software predicted that MACC1 was a direct target of miR‐944. We observed negative regulation of miR‐944 on MACC1 expression, and direct binding between miR‐944 and MACC1 was verified by dual‐luciferase assays in HEK293T cells. Restoration of MACC1 resulted in promoted EMT and metastasis in miR‐944‐overexpressing MGC‐803 cells. Loss of MACC1 abrogated the effects of miR‐944 knockdown on EMT and metastasis of SGC‐7901 cells. We also found that the Met–AKT pathway might be involved in MACC1‐mediated EMT. In conclusion, miR‐944 acts as an inhibitor of EMT and metastasis of GC by targeting MACC1. This study highlights the potential effects of miR‐944 in the prognosis and treatment of GC.

**Abbreviations**
CRC: colorectal cancer
DAPI: 4′,6‐diamidino‐2‐phenylindole
EMT: epithelial–mesenchymal transition
GAPDH: glyceraldehyde 3‐phosphate dehydrogenase
GC: gastric cancer
IF: immunofluorescence
MACC1: metastasis‐associated in colon cancer 1
miRNA: microRNA
NSCLC: non‐small cell lung cancer
TCGA: The Cancer Genome Atlas

Gastric cancer (GC) is the most frequent primary cancer of digestive tract and the second leading cause of cancer‐related death worldwide 1. Although treatment has improved, the metastasis and recurrence of GC compromise the efficiency of new therapies, and the survival of GC patients remains dismal 2. Further investigation of mechanisms involved in GC metastasis and recurrence is required.

MicroRNAs (miRNAs) are small non‐coding RNAs that post‐transcriptionally regulate gene expression by binding the 3′‐untranslated regions (3′‐UTRs) of mRNAs 3. Dysregulated miRNAs contribute to cancer initiation and progression by acting as proto‐oncogenes or tumor suppressor genes 4. miR‐944 functions as one of prognostic miRNAs in cancer tissue from patients operated for pancreatic cancer 5. Furthermore, miR‐944 is identified as one potential driver miRNA in non‐small cell lung cancer (NSCLC) 6, 7. Overexpression of miR‐944 promotes tumorigenesis of NSCLC by targeting suppressor of cytokine signaling 4 (SOCS4) 8. Increased plasma circulation of miR‐944 acts as a potential diagnostic biomarker of squamous cell carcinoma in lung cancer 9. miR‐944 is significantly overexpressed in cervical cancer and promotes proliferation as well as migration and invasion in cancer cells 10. Up‐regulation of miR‐944 is observed in breast cancer patients’ serum and tumor tissues, and it promotes the chemotherapy of breast cancer by targeting BCL2 interacting protein 3 (BNIP3). miR‐944 is identified as being prominently downregulated in exosomes arising from adenocarcinoma of the esophagus 11. Flores‐Pérez *et al*. 12 reported that miR‐944 expression was significantly silenced in clinical specimens and breast cancer cell lines, and miR‐944 promoted cell migration through targeting of siah E3 ubiquitin protein ligase 1 (SIAH1) and protein tyrosine phosphatase type IVA, member 1 (PTP4A1). A recent study reported that the levels of miR‐944 in recurrent colorectal cancer (CRC) patients were evidently lower than those in non‐recurrent cases, suggesting that miR‐944 may function as a tumor suppressive miRNA in CRC 13. However, the clinical significance and biological role of miR‐944 in GC remain largely unknown.

This study showed that miR‐944 underexpression was observed in GC tissues and cells. We also showed that loss of miR‐944 promoted GC cell migration and invasion, and resulted in epithelial–mesenchymal transition (EMT) progression probably by targeting metastasis‐associated in colon cancer 1 (MACC1)–Met–AKT signaling *in vitro*. In conclusion, this work provides the first evidence that miR‐944 is a potential therapeutic target in GC.

## Materials and methods

### Cell culture and transfection

Human GC cell lines (SGC‐7901, MGC‐803, MKN‐28 and BGC‐823) and a normal gastric epithelium cell line (GES‐1) were purchased from the Cell Bank of Shanghai Institute of Cell Biology, Chinese Academy of Medical Science (Shanghai, China). Cells were cultured in DMEM with 10% Gibco fetal bovine serum (Thermo Fisher Scientific, Waltham, MA, USA) with antibiotics (Sigma‐Aldrich, St. Louis, MO, USA) at 37 °C in 5% CO_2_.

Precursor miRNA clones (mimic‐miR‐944), miR‐944 inhibitors (anti‐miR‐944), MACC1 over‐expression plasmid (pcDNA3.1‐MACC1) and corresponding negative control were designed and synthesized by GeneCopoeia (Guangzhou, China). MACC1 siRNA and a scrambled control siRNA were designed and synthesized by Shanghai GenePharma Co., Ltd (Shanghai, China). Cell transfection was performed by using Lipofectamine 2000 (Invitrogen/Thermo Fisher Scientific) according to the supplier's protocol.

### Quantitative real‐time PCR (qRT‐PCR)

Total RNA was extracted from GC cells and tissues with Trizol reagent (Invitrogen/Thermo Fisher Scientific). PrimeScript RT Master Mix (Perfect Real Time) (TaKaRa, Shiga, Japan) was used to assess MACC1, while a poly‐A polymerase‐based First‐Strand Synthesis Kit (TaKaRa) was used for miR‐944 by polyadenylating the total RNA. After reverse transcription, qRT‐PCR was performed by using SYBR Premix E Taq 2 (TaKaRa). MACC1 was normalized to glyceraldehyde 3‐phosphate dehydrogenase (GAPDH) and U6 was used as miR‐944 endogenous control. The primers used for miR‐944 and U6 as well as MACC1 and GAPDH were designed and purchased from Sangon Biotech (Shanghai, China).

### Western blot

Antibodies for western blot analysis were as follows: MACC1 (Abcam, Cambridge, MA, USA), Met (Cell Signaling Technology, Danvers, MA, USA), AKT (Cell Signaling), p‐AKT (Ser473) (Cell Signaling), E‐cadherin (Abcam), N‐cadherin (Abcam), vimentin (Abcam) and GAPDH (G8140, US Biological, Swampscott, MA, USA). The goat anti‐rabbit/mouse secondary antibodies were obtained from Cell Signaling. Two days post‐transfection, total proteins were extracted, followed by quantification with a Pierce BCA protein assay kit (Pierce, Bonn, Germany). Proteins were separated by 10% SDS‐PAGE gels and transferred to poly(vinylidene difluoride) membranes. After blocking, blots were probed with specific antibodies.

### Wound healing assay

GC cells that were transfected with corresponding vectors were seeded in six‐well plates to form the single confluent cell layer. Wounds were made with 100 μL tips in the confluent cell layer; 0 and 24 h after would scratching, the wounds were photographed with a phase‐contrast microscope and wound width determined.

### Migration and invasion assay

We determined the cell migration and invasion capacities by using Transwell chambers of pore size 8 μm (Coring Costar, Cambridge, MA, USA). Twenty‐four hours after transfection, 5 × 10^4^ cells were seeded in the uncoated (migration assay) or 1 : 9 diluted Matrigel‐coated (BD Biosciences, Franklin Lakes, NJ, USA) upper chamber (invasion assay) with 250 μL serum‐free DMEM, while 700 μL DMEM with 10% serum was added in the lower chamber. After 24 h (migration assay) or 48 h (invasion assay), we fixed the cells with paraformaldehyde and the cells in the upper chamber were removed. Cells in the lower chamber were then stained using 0.1% crystal violet solution and photographed.

### Dual‐luciferase reporter assay

Luciferase reporter vector containing the potential binding sequence of the 3′‐UTR of MACC1 was cotransfected with mimic‐miR‐944, mutant‐miR‐944 and corresponding negative control in HEK293T cells in a 96‐well plate. Two days later, a dual‐luciferase reporter assay system (Promega, Madison, WI, USA) was used to measure the alteration of luciferase activity. Firefly luciferase activity was normalized to *Renilla* luciferase activity.

### Immunofluorescence

GC cells were seeded on chamber slides and fixed with 4% paraformaldehyde for 10 min at room temperature. Then, cells were incubated with antibodies against E‐cadherin (Abcam), N‐cadherin (Abcam) or vimentin (Abcam) at 4 °C overnight. Then, the slides were incubated with matched secondary antibodies (Invitrogen/Thermo Fisher Scientific) at room temperature for 1 h. The nuclei of GC cells were stained with 4′,6‐diamidino‐2‐phenylindole (DAPI; Sigma‐Aldrich) at room temperature for 10 min. Fluorescence confocal images were captured using an LSM 5 Pascal laser scanning microscope (Zeiss, Oberkochen, Germany).

### Patients and tissue samples

Forty pairs of human GC and matched adjacent normal gastric tissues were obtained from GC patients undergoing gastrectomy at the Department of Surgical Oncology in Sir Run Run Shaw Hospital, School of Medicine, Zhejiang University. All tissue samples were stored in liquid nitrogen immediately after surgical excision. Patients in the group did not receive any anti‐tumor therapy before surgical excision. All patients were well informed and signed informed consents. The study was conducted in accordance with the Declaration of Helsinki, and the protocol was approved by the Ethics Committee of Zhejiang University.

### Statistical analysis

Data were presented as mean ± SEM and analyzed by prism 5 software (GraphPad Software, Inc., San Diego, CA, USA). Comparison between groups was analyzed using Student's *t* test or ANOVA. Correlation analysis was performed by Spearman's rank correlation test. *P* < 0.05 was considered statistically significant.

## Results

### Loss of miR‐944 promotes the invasion and migration of GC cell lines *in vitro*

The expression of miR‐944 in 40 cases of GC tissue and matched adjacent normal gastric tissue was evaluated by qRT‐PCR. The results showed that the expression of miR‐944 was significantly down‐regulated in GC tissues (*P* < 0.05, Fig. 1A). miRNA quantification data for 100 GC and 10 normal unmatched gastric samples were downloaded from The Cancer Genome Atlas (TCGA) database. Reads per million miRNA mapped values were used to represent miRNA expression levels. Analysis of TCGA miRNA expression data showed significantly lower expression of miR‐944 in GC tumors than in normal gastric tissues (*P* < 0.05, Fig. 1B). Underexpression of miR‐944 was observed in GC cell lines (SGC‐7901, BGC‐823, MKN‐28 and MGC‐803) compared with GES‐1 cells (*P* < 0.05, Fig. 1C). Moreover, we tested the effects of miR‐944 on invasion and migration capacities of GC cells *in vitro*. MGC‐803 cells showed the lowest while SGC‐7901 cells showed the highest level of miR‐944 in all GC cell lines. Accordingly, gain‐ and loss‐of‐function experiments were performed in MGC‐803 and SGC‐7901 cells, respectively. Mimic‐miR‐944 transfection resulted in significant increase of miR‐944 expression in MGC‐803 cells (*P* < 0.05, Fig. 2A). miR‐944 overexpression inhibited migration and invasion abilities in MGC‐803 cells (*P* < 0.05, respectively, Fig. 2B,C), while opposite results were further observed after anti‐miR‐944 transfection in both SGC‐7901 and BGC‐823 cells (*P* < 0.05, Fig. 3). These data disclose the anti‐metastatic role of miR‐944 in GC cells.

**Figure 1:** MiR‐944 is underexpressed in GC tumor tissues and cells. (A) qRT‐PCR was performed to identify the alterative expression of miR‐944 in 40 pairs of human GC and matched adjacent normal gastric tissues. (B) Analysis of TCGA miRNA expression data showing significantly lower expression of miR‐944 in GC tumors (*n* = 100) than in normal gastric tissues (*n* = 10). (C) The differences in expression of miR‐944 between GC cell lines (SGC‐7901, BGC‐823, MKN‐28 and MGC‐803) and a normal gastric epithelium cell line (GES‐1). *P < 0.05.

**Figure 2:** MiR‐944 overexpression inhibits cell migration and invasion in MGC‐803 cells. (A) MGC‐803 cells that were transfected with miR‐944 mimic (50 nm; mimic‐miR‐944) and miRNA scrambled control (50 nm; mimic‐NC) were subjected to qRT‐PCR for miR‐944 expression. (B) Wound healing assays indicated that miR‐944 overexpression inhibited cell migration in MGC‐803 cells. (C) The invasion and migration capacity of MGC‐803 cells were measured by Transwell assays after miR‐944 mimic treatments. *P < 0.05. Scale bar: 100 μm.

**Figure 3:** Loss of miR‐944 facilitates cell migration and invasion in SGC‐7901 and BGC‐823 cells. (A) SGC‐7901 cells that were transfected with miR‐944 inhibitor (200 nm; anti‐miR‐944) and miRNA inhibitor scrambled control (200 nm; anti‐NC) were subjected to qRT‐PCR for miR‐944 expression. (B) Wound healing assays revealed that miR‐944 knockdown promoted cell migration in SGC‐7901 cells. (C) The invasion and migration capacity of SGC‐7901 cells were enhanced as measured by Transwell assays after miR‐944 silencing. *P < 0.05. Scale bar: 100μm. (D) Transwell assays indicated that miR‐944 knockdown facilitated the migration and invasion in BGC‐823 cells. *P < 0.05. Scale bar: 100 μm.

### Underexpression of miR‐944 promotes the EMT process of GC cells

As miR‐944 maintained an anti‐metastasis ability for GC, we then explored the underlying relationship between miR‐944 and EMT. Interestingly, western blotting and immunofluorescence (IF) results indicated that notable gain of epithelial marker (E‐cadherin) and obvious loss of mesenchymal markers (N‐cadherin, vimentin) were detected after miR‐944 restoration in MGC‐803 cells (*P* < 0.05, Fig. 4A,B). Conversely, anti‐miR‐944 decreased the expression of E‐cadherin but increased the levels of N‐cadherin and vimentin in both SGC‐7901 and BGC‐823 cells (*P* < 0.05, Fig. 4C–E). Therefore, our data demonstrate that loss of miR‐944 enhances invasion and migration abilities of GC cells probably by promoting the EMT process.

**Figure 4:** Loss of miR‐944 results in enhanced EMT in GC cell lines. (A) Mimic‐miR‐944 treatment up‐regulated the expression of epithelial marker (E‐cadherin) and resulted in reduced levels of mesenchymal markers (N‐cadherin and vimentin) in MGC‐803 cells. *P < 0.05. (B) The biomarkers of EMT (E‐cadherin and vimentin) in mimic‐miR‐944‐treated GC cell lines were further verified by IF. Scale bar: 20 μm. (C) Decreased expression of E‐cadherin and up‐regulation of N‐cadherin and vimentin were observed in miR‐944‐silenced SGC‐7901 cells. *P < 0.05. (D) Immunostaining of E‐cadherin and vimentin were confirmed by IF in anti‐miR‐944‐treated SGC‐7901 cells. Scale bar: 20 μm. (E) Reduced expression of E‐cadherin and elevated levels of N‐cadherin and vimentin were detected after miR‐944 knockdown by immunoblotting in BGC‐823 cells. *P < 0.05.

### MACC1 is the direct target of miR‐944 in GC

According to the prediction of bioinformatics software (targetscan), MACC1 is considered as one of the candidates with which miR‐944 could bind directly (Fig. 5A). We tested whether miR‐944 could participate in the modulation of MACC1. The gain‐ and loss‐of‐function experiments of miR‐944 in GC cells showed that the expression of MACC1 protein could be negatively regulated by miR‐944 (*P* < 0.05, Fig. 5B). Moreover, miR‐944 overexpression obviously inhibited luciferase activity of the reporter with 3′‐UTR sequence of MACC1 (*P* < 0.05, Fig. 5C), but mutant miR‐944 showed no significant effect on luciferase activity (Fig. 5C). The levels of MACC1 mRNA were detected by qRT‐PCR in 40 samples of GC tissues. Spearman's rank correlation test revealed that the levels of MACC1 were inversely correlated with miR‐944 expression in GC tissues (*r* = −0.673, *P* < 0.05, Fig. 5D). Hence, miR‐944 down‐regulates the expression of MACC1 in GC cells by binding to its 3′‐UTR sequence directly.

**Figure 5:** MACC1 is the direct target of miR‐944 in GC cells. (A) The potential miR‐944 binding site in 3′‐UTR sequence of MACC1. The mutant site designed for miR‐944 is shown underlined. (B) The regulatory role of miR‐944 on MACC1 expression in GC cell lines was determined by western blot analysis. *P < 0.05. (C) HEK293T cells were cotransfected with mimic‐NC/mimic‐miR‐944/mutant‐miR‐944 and luciferase reporters containing 3′‐UTR of MACC1 sequence. miR‐944 overexpression decreased the luciferase activity of MACC1 3′‐UTR, while mutant‐miR‐944 showed no significant effect on the luciferase activity. *P < 0.05. (D) An inverse correlation between the levels of miR‐944 and MACC1 mRNA expression was observed in 40 cases of GC tissues.

### Re‐expression of MACC1 reverses the anti‐metastatic role of miR‐944 in GC cells

We next determined whether re‐expression of MACC1 would rescue the effects of mimic‐miR‐944 in GC cells. As expected, restoration of MACC1 rescued the prohibited effect of mimic‐miR‐944 on MACC1, as well as EMT‐related biomarkers (E‐cadherin, N‐cadherin and vimentin) (*P* < 0.05, Fig. 6A). Decreased migratory and invasive abilities caused by mimic‐miR‐944 were subsequently abolished by MACC1 over‐expression in GC cells (*P* < 0.05, respectively, Fig. 6B,C). Furthermore, loss of MACC1 abrogated the effects of miR‐944 knockdown on EMT events and metastasis of SGC‐7901 cells (*P* < 0.05, Fig. 6D,E). Hence, these results further confirm that loss of miR‐944 promotes EMT and metastasis of GC by targeting MACC1.

**Figure 6:** Restoration of MACC1 reversed miR‐944‐inhibited EMT process in GC cells. (A) MGC‐803 cells that were previously transfected with miR‐944 mimic were transfected with control vector (pcDNA3.1‐NC) and pcDNA3.1‐MACC1, respectively. The expressions of MACC1 and EMT biomarkers in mimic‐miR‐944 transfected MGC‐803 cells was determined by performing immunoblotting after MACC1 overexpression. *P < 0.05. (B) MACC1 restoration facilitated the migration of miR‐944‐overexpressing MGC‐803 cells. (C) Forced expression of MACC1 reversed the inhibitory effects of miR‐944 on migration and invasion capacity of MGC‐803 cells. *P < 0.05. Scale bar: 100μm. (D) SGC‐7901 cells that were previously transfected with miR‐944 inhibitor were transfected with scrambled control siRNA (siNC) and MACC1 siRNA (siMACC1), respectively. The expressions of MACC1 and EMT biomarkers were detected by western blotting. *P < 0.05. (E) Loss of MACC1 abolished the promoting effects of miR‐944 silencing on SGC‐7901 cell migration and invasion. *P < 0.05. Scale bar: 100 μm.

### The Met–AKT signaling axis may be involved in the miR‐944–MACC1‐mediated EMT

As previous studies have identified that activated Met–AKT signaling could promote the EMT process 14, we next determined whether the Met–AKT signaling axis was involved in the miR‐944–MACC1‐mediated EMT process. Interestingly, we found that the ratio of Met and of phosphoryated AKT were notably decreased in the miR‐944 overexpression group, while MACC1 over‐expression led to increased activity of the Met–AKT signaling pathway (*P* < 0.05, Fig. 7). Therefore, these results indicates that the Met–AKT signaling axis may be involved in the miR‐944–MACC1‐mediated EMT process.

**Figure 7:** The Met–AKT signaling axis is involved in the miR‐944–MACC1‐mediated EMT. The activity of the Met–AKT pathway was suppressed by mimic‐miR‐944 treatment with down‐regulation of Met and p‐AKT as examined by western blot analysis. MACC1 restoration abrogated the inhibitory effects of miR‐944 on the activity of Met–AKT signaling. *P < 0.05.

## Discussion

Recent studies have demonstrated that miRNAs are involved in tumor initiation and progression as either oncogenes or tumor suppressors by negatively regulating downstream targets 15, 16, 17, and therefore identifying these miRNAs provides novel insight for the diagnosis and therapy of GC patients 16, 18. Here, our data indicated that underexpressed miR‐944 was common in GC tissues, which was consistent with the results of Christensen *et al*. for CRC 13. Moreover, the expression of miR‐944 was intensively reduced in GC cell lines compared with a normal gastric epithelium cell line (GES‐1). Although great effort has been put into the study of miR‐944 in tumor cell growth and apoptosis 7, 10, the roles of miR‐944 in the modulation of the EMT process remain largely unknown. In our present study, gain‐ and loss‐of‐function methods were used to determine the functional roles of miR‐944 in EMT. After restoration of miR‐944, up‐regulated expression of E‐cadherin (an epithelial marker) and suppressed expression of N‐cadherin and vimentin (mesenchymal markers) were detected, accompanying inhibited cell invasion and migration abilities in MGC‐803 cells. The opposite data were obtained with anti‐miR‐944 treatment in both SGC‐7901 and BGC‐823 cells. These results demonstrate that miR‐944 serves as a tumor suppressor by suppressing EMT in GC.

MACC1 is considered to play a vital role in the pro‐cancer process. In colon cancer cells, MACC1 promotes proliferation, invasion and hepatocyte growth factor‐induced scattering 19. Researchers have found that MACC1 is significantly up‐regulated in GC tissues 20 and promotes tumor cell proliferation and invasion 21. Moreover, it has also been found that MACC1 is associated with aggressive clinicopathological features of GC 22. In this study, we found that MACC1 is a direct target of miR‐944. Notably, re‐expression of MACC1 rescued miR‐944 inhibition of the EMT process and tumor metastasis, while loss of MACC1 abrogated miR‐944 silencing‐induced EMT events and tumor metastasis. These results demonstrate that miR‐944 inhibits the EMT process and GC metastasis probably by targeting MACC1.

Met–AKT signaling plays vital roles in the modulation of carcinogenesis. In papillary thyroid carcinoma, the blockage of the Met–AKT pathway inhibits cell proliferation and induces apoptosis 23. Activation of the Met–AKT pathway is engaged in sorafenib and apoptosis resistance in GC 24, 25. It is also reported that miR‐338‐3p inhibits EMT in GC cells by targeting zinc finger E‐box binding homeobox 2 (ZEB2) and MACC1–Met–Akt signaling 14. Hence, we investigated the effect of MACC1 restoration on the Met–AKT signaling pathway in order to elucidate the potential mechanism of MACC1‐mediated EMT. As expected, the levels of Met and phosphorylated AKT were downregulated in miR‐944‐overexpressing cells and they were up‐regulated in the pcDNA3.1‐MACC1 group. These results indicate that the Met–AKT signaling pathway may be involved in the miR‐944–MACC1‐mediated EMT process and tumor metastasis. However, further investigations are needed to reach a firm conclusion.

To conclude, the underexpression of miR‐944 creates a milieu of EMT facilitation that plays a promoting role in GC progression. A mechanism by which underexpressed miR‐944 promotes EMT and tumor metastasis by targeting MACC1 plays an important role in this process. This finding will improve understanding of the EMT progression mechanism and provide novel targets for the molecular treatment of GC.

## Conclusions

Dysfunction of miRNAs has been implicated in the initiation and progression of human cancers. miR‐944 was previously found to be a cancer‐related miRNA, but the clinical significance and biological function of miR‐944 remain poorly known in GC. Here, we presented evidence that the miR‐944 level in GC tissues was notably reduced compared with matched non‐cancerous specimens. Accordingly, the levels of miR‐944 were obviously down‐regulated in GC cells compared with GES‐1 cells. Ectopic expression of miR‐944 in MGC‐803 cells prominently inhibits the migration and invasion of tumor cells, while miR‐944 knockdown increased these behaviors of both SGC‐7901 and BGC‐823 cells. Mechanically, miR‐944 exerted an anti‐metastatic function by suppressing EMT and MACC1 abundance in GC cells. Herein, MACC1 was found to be a downstream molecule of miR‐944 in GC. Furthermore, restoration of MACC1 expression could abrogate the anti‐metastatic effects of miR‐944 on MGC‐803 cells with enhanced EMT as well as cell migration and invasion. Loss of MACC1 abrogated the effects of miR‐944 knockdown on the EMT process and metastasis of SGC‐7901 cells. Notably, the Met–AKT signaling axis might be involved in the role of the miR‐944–MACC1‐mediated EMT process. Altogether, miR‐944 potentially acts as a drug target for GC patients.

## Author contributions

TP, XY, JS, CQ and LW carried out the cell biology and molecular biology experiments, participated in the sequence alignment and drafted the manuscript. TP and WC participated in the design of the study and performed the statistical analysis. WC conceived of the study, and participated in its design and coordination and helped to draft the manuscript. All authors read and approved the final manuscript.
